The article "Training a Feedforward Neural Network Using Hybrid Gravitational Search Algorithm with Dynamic Multiswarm Particle Swarm Optimization" was retracted in 2024. Reasons: signs of a paper mill; suspected computer-generated content; unreliable results or conclusions; concerns about the data.

# Training a Feedforward Neural Network Using Hybrid Gravitational Search Algorithm with Dynamic Multiswarm Particle Swarm Optimization

**DOI:** 10.1155/2022/2636515

**Published:** 2022-05-30

**Authors:** Arfan Ali Nagra, Tahir Alyas, Muhammad Hamid, Nadia Tabassum, Aqeel Ahmad

**Affiliations:** ^1^Department of Computer Science, Lahore Garrison University, Lahore 54000, Pakistan; ^2^Department of Statistics and Computer Science, University of Veterinary and Animal Sciences, Lahore 54000, Pakistan; ^3^Department of Computer Science, Virtual University of Pakistan, Lahore 54000, Pakistan; ^4^University of Chinese Academy of Sciences (UCAS), Beijing, China

## Abstract

One of the most well-known methods for solving real-world and complex optimization problems is the gravitational search algorithm (GSA). The gravitational search technique suffers from a sluggish convergence rate and weak local search capabilities while solving complicated optimization problems. A unique hybrid population-based strategy is designed to tackle the problem by combining dynamic multiswarm particle swarm optimization with gravitational search algorithm (GSADMSPSO). In this manuscript, GSADMSPSO is used as novel training techniques for Feedforward Neural Networks (FNNs) in order to test the algorithm's efficiency in decreasing the issues of local minima trapping and existing evolutionary learning methods' poor convergence rate. A novel method GSADMSPSO distributes the primary population of masses into smaller subswarms, according to the proposed algorithm, and also stabilizes them by offering a new neighborhood plan. At this time, each agent (particle) increases its position and velocity by using the suggested algorithm's global search capability. The fundamental concept is to combine GSA's ability with DMSPSO's to improve the performance of a given algorithm's exploration and exploitation. The suggested algorithm's performance on a range of well-known benchmark test functions, GSA, and its variations is compared. The results of the experiments suggest that the proposed method outperforms the other variants in terms of convergence speed and avoiding local minima; FNNs are being trained.

## 1. Introduction

In computational intelligence, neural networks (NNs) are one of the most advanced creations. Neurons in the human brain are often employed to solve categorization problems. The basic notions of NNs were first articulated in 1943 [1]. Feedforward [2], Kohonen self-organizing network [3], radial basis function (RBF) network [4], recurrent neural network [5], and spiking neural networks [6] are some of the NNs explored in this paper.

Data flows in one direction via the networks in FNN. In recurrent NNs, data is shared in two directions between the neurons. Regardless of the variances amongst NNs, they all learn in the same way. The ability of a NN to learn from experience is referred to as learning. Similar to real neurons, artificial neural networks (ANN) [7, 8] have been constructed with strategies to familiarise themselves with a set of specified inputs. In this context, there are two types of learning: supervised [9] and unsupervised [10]. The NN is given feedback from an outside source in the first way. The NN familiarises itself with inputs without any external feedback in unsupervised learning. Feedforward Neural Networks with multilayer [11] have recently become popular. In practical applications, FNNs with several layers are the most powerful neural networks. Multilayer FNNs have been shown to be fairly accurate for both continuous and discontinuous functions [12]. Many studies find that learning is an important aspect of any NN. For the standard [13] or enhanced [14], the leading applications have employed the Backpropagation (BP) algorithm as the training. strategy for FNNs. Backpropagation (BP) is a gradient-based approach with drawbacks such as delayed convergence [15] and the ability to become trapped in local minima.

The article "Training a Feedforward Neural Network Using Hybrid Gravitational Search Algorithm with Dynamic Multiswarm Particle Swarm Optimization" was retracted in 2024. Reasons: signs of a paper mill; suspected computer-generated content; unreliable results or conclusions; concerns about the data.

Various optimization approaches have already been applied simulated annealing, for example, which may be used to train FNNs (SA) [16], particle swarm optimization (PSO) algorithms [17], Magnetic Optimization Algorithm (MOA) [18], GG-GSA [19], and PSOGSA [20]. Genetic Algorithm (GA) [21], Differential Evolution (DE) [22], Ant Colony Optimization (ACO) [23], Artificial Bee Colony (ABC) [24], Hybrid Central Force Optimization and Particle Swarm Optimization (CFO-PSO) [25], Social Spider Optimization algorithm (SSO) [26], Chemical Reaction Optimization (CRO) [27], Charged System Search (CSS) [28], Invasive Weed Optimization (IWO) [29], and Teaching-Learning Based Optimization (TLBO) trainer [30] are some of the most popular evolutionary training algorithms. According to [31, 32], PSO and GSA are one of the best optimization techniques for eliminating both issues of slow convergence rate and trap in local optima. Recently, hybrid methods had been introduced to overcome the weakness of slow convergence [33, 34]. Most of the previous algorithms fail to reach the minimal selection; the hybrid gravitational search algorithm with social ski-driver- (GSA-SSD-) based model has been introduced to overcome the convergence problem [35].

To overcome these weaknesses, GSADMSPSO [36] is used as a Feedforward Neural Network (FNN) as a new approach to examine the algorithm's efficiency and reduce the difficulties of minima in the immediate vicinity trapping and slow steady convergence. Algorithms for evolutionary learning GSADMSPSO distribute the primary population of masses into smaller subswarms, according to the suggested algorithm, and also stabilize them by offering a fresh neighborhood plan [37]. At this time, each agent (particle) increases its position and velocity by using the suggested algorithm's global search capability. The fundamental concept is to combine GSA's ability with DMSPSO's to improve the performance of a given algorithm's exploration and exploitation [38]. The suggested method's performance is compared to that of GSA and its variants using well-known benchmark test functions [39, 40]. The experimental results show that in terms of avoiding local minima and accelerating convergence, the proposed approach beats existing FNN training variations. The following is the order of this paper's remaining sections: Section 1 introduces the basic concept of GSA. The dynamic multiswarm particle swarm optimization and gravitational search approach are discussed in Section 2; then, in Section 3, we go over the GSADMSPSO methodology in depth. The experiment's findings are provided in Section 4.  Section 5 discusses contrast analysis. In the concluding section, the findings are given.

The article "Training a Feedforward Neural Network Using Hybrid Gravitational Search Algorithm with Dynamic Multiswarm Particle Swarm Optimization" was retracted in 2024. Reasons: signs of a paper mill; suspected computer-generated content; unreliable results or conclusions; concerns about the data.

## 2. Related Work

### 2.1. Multilayer Perceptron with Feedforward Neural Network

The connections of FNNs between the neurons are unidirectional and one-way. In neural networks [2], neurons are in parallel layers. The first layer is the input layer, the second layer is the concealed layer, and the last layer is the output layer.  Figure 1 shows an example of a FNN using MLP.

The output of a given data has been calculated in step by step procedure [18]: the average sum of weight in input is calculated in

(1) $$\begin{array}{c} s_{j}=\overset{n}{\underset{i=1}{\sum }}\left(W_{ij}X_{i}\right)-\theta_{j},\;j=1,2,\cdots ,h. \end{array}$$

The hidden layer values are calculated in

(2) $$\begin{array}{c} s_{j}=\text{sigmoid}\left(s_{j}\right)=\frac{1}{1+\exp\left(-s_{j}\right)},\;j=1,2,\cdots ,h. \end{array}$$

The output MSE and accuracy have been calculated in

(3) $$\begin{array}{c} \;O_{k}=\overset{h}{\underset{j=1}{\sum }}\left(wjk.s_{j}\right)-\theta^{\prime },\;k=1,2,\cdots ,m, \end{array}$$

(4) $$\begin{array}{c} O_{k}=\text{sigmoid}\left(O_{k}\right)=\frac{1}{1+\exp\left(-O_{k}\right)},\;j=1,2,\cdots ,m. \end{array}$$

From input, the output of MLPs has been observed with the help of biases and weights in equations (1) to (4).

### 2.2. Gravitational Search Algorithm

The typical GSA is a newly projected search algorithm. GSA firstly initializes the positions of *N* agents randomly, shown as

(5) $$\begin{array}{c} X_{i}=\left(x_{i}^{1},\cdots ,x_{i}^{d},\cdots ,x_{i}^{D}\right) \end{array}$$

for *i* = 1, 2, ⋯, *N*, where *D* is the dimension index of the search space and *x*_*i*_^*d*^ represents the *i*^th^ agent in the *d*^th^ dimension:

(6) $$\begin{array}{c} q_{i}\left(t\right)=\frac{{\text{fit}}_{i}-\text{worst}\left(t\right)}{\text{best}\left(t\right)-\text{worst}\left(t\right)}, \end{array}$$

(7) $$\begin{array}{c} M_{i}\left(t\right)=\frac{q_{i}\left(t\right)}{\sum_{j=1}^{N}q_{j}\left(t\right)}, \end{array}$$

where fit_*i*_(*t*) and *M*_*i*_(*t*) represent the fitness and best(*t*) and worst(*t*) are defined in the following equations:

(8) $$\begin{array}{c} \text{best}\left(t\right)=\min_{j\epsilon \left\{1,\cdots ,N\right\}}{\text{fit}}_{j}\left(t\right), \end{array}$$

(9) $$\begin{array}{c} \text{worst}\left(t\right)=\max_{j\epsilon \left\{1,\cdots ,N\right\}}{\text{fit}}_{j}\left(t\right). \end{array}$$

The force acting on *i*^th^ agent from *j*^th^ agent is as follows:

(10) $$\begin{array}{c} f_{ij}^{d}\left(t\right)=G\left(t\right)\frac{M_{i}\left(t\right)\times M_{j}\left(t\right)}{R_{i,j+\epsilon }}\left(x_{j}^{d}\left(t\right)-x_{i}^{d}\left(t\right).\right. \end{array}$$

*G*(*t*) is a function of the iteration time:

(11) $$\begin{array}{c} G\left(t\right)=G_{0}e^{-\alpha t/T}, \end{array}$$

where *G*_0_ is the initial value, *α* is a shrinking parameter, and *T* represents the maximum number of iterations:

(12) $$\begin{array}{c} {F_{i}}^{d}\left(t\right)=\underset{j\in K\text{best},j\neq i}{\sum }{\mathrm{rand}}_{j}F_{ij}^{d}\left(t\right), \end{array}$$

where *K*best is the set of the first *K* agents with the biggest mass; the acceleration of the *i*^th^ agent is calculated as follows:

(13) $$\begin{array}{c} a_{i}^{d}\left(t\right)=\frac{{F_{i}}^{d}\left(t\right)}{M_{i}\left(t\right)}. \end{array}$$

Further velocity is updated using the following equation:

(14) $$\begin{array}{c} v_{i}^{d}\left(t+1\right)={\mathrm{rand}}_{i}\times v_{i}^{d}\left(t\right)+a_{i}^{d}\left(t\right), \end{array}$$

(15) $$\begin{array}{c} x_{i}^{d}\left(t+1\right)=x_{i}^{d}+v_{i}^{d}\left(t+1\right). \end{array}$$

By summing up the equations, acceleration can also be written as

(16) $$\begin{array}{c} a_{i}^{d}\left(t\right)=\underset{j\in K\text{best},j\neq i}{\sum }{\mathrm{rand}}_{j}\times M_{j}\left(t\right)\frac{G\left(t\right)}{R_{ij}\left(t\right)+\epsilon }\left(x_{j}^{d}\left(t\right)-x_{i}^{d}\left(t\right)\right). \end{array}$$

The article "Training a Feedforward Neural Network Using Hybrid Gravitational Search Algorithm with Dynamic Multiswarm Particle Swarm Optimization" was retracted in 2024. Reasons: signs of a paper mill; suspected computer-generated content; unreliable results or conclusions; concerns about the data.

### 2.3. The Hybrid GSABP Algorithm

In the optimization problems, there are a lot of local minima. The hybrid method final results reflect the aptitude of the algorithm in overcoming local minima and attaining a close global optimum [36]. The error of FNN is often large in the initial period of the training process. For solving real-world and complex optimization problems, one of the most well-known methods is the gravitational search algorithm (GSA). The gravitational search technique suffers from a slow convergence rate and weak local search capabilities while solving complicated optimization problems. The BP algorithm has a strong ability to search local optimum, but its ability to search global optimum is weak. The hybrid GSABP is proposed to combine the global search ability of GSA with the local search ability of BP. This combination takes advantage of both algorithms to optimize the weights and biases of the FNN.

## 3. The Proposed Hybrid Algorithm

The main concern to hybridize the algorithm is to maintain the constancy between exploration and exploitation. In the initial iterations, it is achieved step size of agents. In the final iterations, it is very difficult to avoid the global optima. Then, in the later iteration, the fitness focus is on small step size for exploitation. For better performance and to solve the problem of early convergence, a hybrid technique is adopted. In final iterations, we have a problem of slow exploitation and deterioration. Weights are used to assess fitness function in GSA. As a result, fit masses are seen as slow-moving, hefty items.

Then, at first iterations, particles ought to travel across the scope of the search. After that, they have found a good answer; they must wrinkle around it in order to obtain the most effective solution out of it. In GSA, the masses get heavier. Because masses swarm around a solution in the later stages of iterations, their weights are virtually identical. Their gravitational forces are about equal in intensity, and they fascinate each other. As a result, they are unable to travel rapidly to the best answer. A variety of issues have been faced by GSA. The algorithm that has been presented has the capacity to overcome the challenges that GSA has had to deal with. As a result, in this paper, GSADMSPSO proposes a neighborhood approach with dynamic multiswarm (DMS).

In the first iteration, the proposed technique promotes exploration, and in the final iteration, it prioritizes exploitation. The proposed approach initially works on masses of agents in the first phase. Because the agent's weight fitness is poor, it will not be able to achieve peak performance and to look into the search area. Agents that are light in weight can be used; heavy-weight agents, on the other hand, can be chosen to utilise their surroundings using neighborhood strategy. As a consequence, a dynamic multiswarm (DMS) is used, along with a novel neighborhood strategy, as illustrated in the equation below:

(17) $$\begin{array}{c} m_{i}\left(t\right)=\left\{\frac{0.9*{\text{fit}}_{i}}{{\text{best}}_{i}\left(t\right)-{\text{worst}}_{i}\left(t\right)}\;\mathrm{mod}\left({\text{fit}}_{j}\right)=0\right.,\text{then regroup the subswarm}, \end{array}$$

where fit_*i*_(*t*) indicates the fitness value of the agent_*i*_ and worst_*i*_ (*t*) and best_*i*_(*t*) are defined as follows:

(18) $$\begin{array}{c} \text{best}\left(t\right)={\text{low}}_{j\epsilon \text{ regroup of swarms}}{\text{fit}}_{i}\left(t\right), \end{array}$$

(19) $$\begin{array}{c} \text{worst}\left(t\right)={\text{high}}_{j\epsilon \text{ regroup of swarm}}{\text{fit}}_{i}\left(t\right). \end{array}$$

The swarm is divided into several subswarms according to equation (17), and each agent's neighbors can attract it by smearing the gravitational pull on it. They use their own members to look for higher placements in the search area. The subswarms, on the other hand, are dynamic, and a regrouping schedule is frequently used to reorganize them, which is a periodic interchange of information. Through an arbitrary regrouping timetable, agents from various subswarms are rebuilt into a new configuration. As a result, DMS can choose the neighbors with the shortest distance. These neighbors called an agent is agent_*i*_. As a result, each component impacts the agent's ability to attract another swarm agent. The DMS has defined the worst and best agent_*i*_. In the last iteration, the global lookup capability of the DMS PSO algorithm was employed, and equations (20) and (21) are utilised to update the individual's location and velocity:

(20) $$\begin{array}{c} v_{i}^{t+1}=wv_{i}^{t}+c_{1}^{\prime }r_{1}a_{i}^{d}\left(t\right)+c_{2}^{\prime }r_{2}\left(g\text{best}-x_{i}\left(t\right)\right), \end{array}$$

(21) $$\begin{array}{c} x_{i}^{t+1}=x_{i}^{\text{t}}+v_{i}^{t+1}, \end{array}$$

where *V*_*i*_ (*t*) is the velocity at which agent_*i*_*c*_1_ and *c*_2_ are accelerating coefficients at iteration *t*. *r*_1_ select a number between 0 and 1 at random which is *r*_2_. The first part is similar to GSA's, with a focus on mass research. The second element is in charge of enticing people to the best crowds thus far. Each mass's distance between you and the best mass is computed using *g*best − *x*_*i*_(*t*) a random percentage of the ultimate force aimed towards the most advantageous mass.

The article "Training a Feedforward Neural Network Using Hybrid Gravitational Search Algorithm with Dynamic Multiswarm Particle Swarm Optimization" was retracted in 2024. Reasons: signs of a paper mill; suspected computer-generated content; unreliable results or conclusions; concerns about the data.

Set the parameters of the algorithm; *N* is the total number of particles, including the total number of particles. In the suggested approach, the amount of times you have iterated is *t*, *G*0 is the gravitational constant, and *a* is the decreasing coefficient. Create populations at random. The particle's location vector is set as *X*_*i*_ = (*x*_1,_*x*_2_, *x*_3_, ⋯, *x*_*n*_); the velocity is initialized as *v*_*i*_ = (*v*_*i*1,_*v*_*i*2_, *v*_*i*3_, ⋯,*v*_in_)^*t*^; the particles are divided into the global best value for numerical subswarms *g*best and the ideal value for each individual *p*best. Eventually, using the formula below, calculate every person's fitness value. Then, using each individual's fitness value, calculate it and keep track of the optimum spot *g*best, constant of gravitation, and the forces that result from it, which are known. At each cycle, the best solution found so far should be updated. Once the accelerations have been calculated and the best solution has been updated, using the DMS PSO algorithm's global search capability, all agents' velocities may be computed using equation (20). Finally, agents' positions are revised as follows (equation (21)). The procedure comes to an end when an end condition is met. The proposed method's general phases are shown in Figure 2.

Because of the dynamic multiswarm nature of our suggested strategy, each agent may examine the best option, and the masses are given access to a kind of local intelligence. In comparison to existing GSA versions, the proposed technique has the potential to offer better outcomes. The efficiency of the proposed methodology is examined in the next part using a variety of static, dynamic, and real-time issues.

## 4. GSADMSPSO for Training FNNs

The proposed approach of each search agent consists of three parts for the training of FNN: The first section discusses the biases; the second section contains the weights that connect the last component comprising the weights that link the hidden layer nodes to the output layer and the input layer nodes to the hidden layer. This section describes the proposed GSADMSPSO method for training a single layer MLP. The proposed FNNGSADMSPSO is used to reduce error and improve accuracy for correct weights and biases. Equations are used to generate output from the input in the FNN model (1–4). The weight and bias values were used in the first stage of the proposed methodology.

Equation (9) states that the error is calculated using the fitness function. Neural network learning is the process of iteratively reducing the cost function. At each iteration, the application weights and biases at FNN have been changed resulting in cost reduction. The suggested FNNGSADMSPSO method can be described as follows:

1. A population is randomly created. It is in charge of a collection of weights and bias values
2. For assessment, the MSE criteria are employed. It is chosen as the best fitness function after being calculated for each iteration on a given training dataset
3. To create a new solution, the best position and best global values are updated
4. The number of iterations during which the global solution's best fitness value was obtained remains unaltered which is tracked using a counter
5. During the iterations, to create a better population, the places with the worst fitness values are determined. The values of their fitness are calculated and compared to prior positions. If the opposite position has a higher fitness value, it will be introduced into the population and assigned to position 7, else it will be assigned to position 6
6. The proposed GSADMSPSO is used to indicate their new positions for updated positions that are not as good as their actual positions
7. The procedure returns to step 2 after creating a new population. The process is continued until the desired number of generations is reached
8. Finally, the best answer is supplied to FNN, and the test data is utilised to evaluate its performance

The article "Training a Feedforward Neural Network Using Hybrid Gravitational Search Algorithm with Dynamic Multiswarm Particle Swarm Optimization" was retracted in 2024. Reasons: signs of a paper mill; suspected computer-generated content; unreliable results or conclusions; concerns about the data.

### 4.1. Fitness Function

The MLP receives the weight and bias matrices and the fitness worth of each option. The solution is calculated using the mean squared error (MSE). The fitness function of suggested algorithms is defined as MSE, which is stated in equation (9):

(22) $$\begin{array}{c} \text{MSE}=\frac{1}{N}\overset{n}{\underset{i=1}{\sum }}{\left(c-o\right)}^{2}, \end{array}$$

where *n* is the number of training samples, *o* denotes the predicted values of the neural network, and *c* denotes the class names. The classification accuracy criteria, aside from the MSE requirement, are used to evaluate MLP's classification performance on the new dataset, which is determined as the following: *Z* is the sample size in the test dataset and *N* is the number of samples successfully classified by the classifier:

(23) $$\begin{array}{c} \text{Accuracy}=\frac{\sim Z\;}{Z}. \end{array}$$

The first approach is used to apply GSA, PSOGSA, GSADMSPSO, and GG-GSA on a FNN in this study. This indicates that the FNN's structure is fixed; GSA, PSOGSA, GSADMSPSO, and GG-GSA select a set of weights and biases that give the FNN the least amount of inaccuracy.

## 5. Results and Discussions

On 16 standard classification datasets, the proposed technique for FNN training is assessed in terms of its effectiveness using the UCI Machine Learning repository [41] which is represented in Table 1. And for three-bit parity, the suggested algorithm's skills in training FNNs are compared using benchmark problems, which are shown in Table 2. It is conceivable that every particle in this issue is randomly started in the [0, 1] range. The gravitational constant (*G*0) is one in FNNGSA, whereas it is set to 20. Particles' initial velocities are arbitrarily created in the range [0, 1], and for each particle, at the start, the acceleration and mass parameters are both set to zero. In FNNPSOGSA, *c*_1_ and *c*_2_ are both set to 1, and the beginning velocities of the agents are generated at random in the range [0,1], and *w* declines linearly from 0.9 to 0.4. In FNNGG-GSA, the gravitational constant (*G*0) is set to 1, while the value is adjusted to 20. Particles' initial velocities are created arbitrarily in the range [0,1], and the initial acceleration and mass values for each particle are set to 0. When *c*_1_ and *c*_2_ are both set to 1, *w* for FNNGSADMSPSO reduces linearly from 0.9 to 0.4, and the agents' beginning velocities are produced at random in the range [0, 1].

The article "Training a Feedforward Neural Network Using Hybrid Gravitational Search Algorithm with Dynamic Multiswarm Particle Swarm Optimization" was retracted in 2024. Reasons: signs of a paper mill; suspected computer-generated content; unreliable results or conclusions; concerns about the data.

### 5.1. The XOR Issue with *N* Bits of Parity

With *N* bits of parity, the XOR problem arises. The *N* bits' parity problem is a well-known nonlinear benchmark problem. The goal is to count how many “1's” are in the input vector. The input vector's XOR result should be reimbursed. The output is “1” if the input vector has an odd number of “1's.” The output is “0” if the input vector has an even number of “1's.”

For three bits, Table 1 shows the problem's inputs and intended outputs: We cannot solve the XOR problem in a linear fashion without hidden layers, and we cannot solve it with a FNN either (perceptron). To solve this problem, we compare a FNN with the structure 3‐*S*‐1, where *S* is the number of hidden nodes, to FNNs with *S* = 5, 6, 7, 8, 9, 10, 11, 13, 15, 20, and 30 in this section.

### 5.2. Comparison with Other Techniques through Parity Problem with Three Bits (3-Bit XOR)

On the suite of three-bit parity problem (3-bit XOR) benchmark functions, GSADMSPSO was compared to other common GSA variations to assess its performance. The suggested method was compared to GSA, PSOGSA, and GG-GSA. Variants were applied to the three-bit parity problem (3-bit XOR) mentioned in Table 2 in this section.  Table 3 displays the average, best, and standard deviation of the Best Square Error (MSE) for all training samples over 30 distinct trials. According to a *t*-test with a significance level of 5%, the bold values represent the best response. When compared to the other algorithms, GSADMSPSO produced the best results. The SIW-APSO-LS gives the best accuracy, according to the results. GSA, GG-GSA, PSOGSA, and Figure 3 depict GSADMSPSO convergence curves based on MSE averages for all training samples throughout 30 different runs. The convergence curves for FNN with *S* = 5, 9, 13, and 30 are shown in Figures 4(a)–(d). These results show that FNNPSOGSA seems to have the best FNN convergence rate.

The article "Training a Feedforward Neural Network Using Hybrid Gravitational Search Algorithm with Dynamic Multiswarm Particle Swarm Optimization" was retracted in 2024. Reasons: signs of a paper mill; suspected computer-generated content; unreliable results or conclusions; concerns about the data.

### 5.3. Comparison with Other Techniques through Standard Classification Datasets

Many experiments were conducted in order to connect the results of the GSADMSPSO technique with that of the GSA, GG-GSA, and GSADMSPSO methods, and Table 4 shows the PSOGSA feature selection techniques and outcomes in terms of averages, bests, and standard deviations. According to a *t*-test with a significance level of 5%, the bold values in the tables represent the best practicable solution for the difficulties.

On various datasets, Table 4 provides the average classification accuracy of the four methods. As shown in Table 4, in 12 datasets, the suggested approach achieves the highest classification accuracy. In terms of average classification accuracy, GG-GSA outperforms the other two datasets.

According to these findings, the suggested technique beats the competition in datasets with less input parameters. The suggested algorithm's improved exploration and exploitation capacity is the cause for its high performance.  Figure 4 shows the convergence curves of different algorithms based on averages of MSE for all training samples over 30 independent runs in a 3-bit XOR problem.

The results show that the proposed method is very much successful in FNN training, because there is a balance between exploration and exploitation; this is the case. GSADMSPSO shows decent exploration since all search agents collaborate in updating a search agent's location. Because of the inherent social component of PSO, GSADMSPSO's exploitation is highly accurate, resulting in rapid convergence. GSADMSPSO can prevent local optima and improve search space convergence.

## 6. Conclusion

Many real-world issues can be solved using gravity-based search techniques. As a result, in this paper, a unique GSADMSPSO is suggested. Using GSA, PSOGSA, GG-GSA, and GSADMSPSO, four novel training algorithms dubbed FNNGSA, FNNPSOGSA, FNNGG-GSA, and FNNGSADMSPSO are introduced and examined in this paper. The benchmark tasks were 3-bit XOR, function, and 16 conventional categorization problems, and the results show that the suggested approach is quite successful in FNN training, because there is a decent trade-off between exploration and exploitation; this is the case. GSADMSPSO exhibits good exploration since all search agents collaborate in updating a search agent's location. Because of the inherent social component of PSO, GSADMSPSO's exploitation is highly accurate, resulting in rapid convergence. GSADMSPSO can prevent local optima and improve search space convergence.

The article "Training a Feedforward Neural Network Using Hybrid Gravitational Search Algorithm with Dynamic Multiswarm Particle Swarm Optimization" was retracted in 2024. Reasons: signs of a paper mill; suspected computer-generated content; unreliable results or conclusions; concerns about the data.

## Figures and Tables

**Figure 1:** One hidden layer in a multilayer perceptron.

**Figure 2:** Flow chart of a GSADMSPSO.

**Figure 3:** The framework of the proposed method.

**Figure 4:** Convergence curves of different algorithms based on averages of MSE for all training samples over 30 independent runs in a 3-bit XOR problem. (a–d) Are the convergence curves for FNNs with *S* = 5, 9, 13, and 20, respectively.

**Table 1:** UCI has compiled a list of real-world datasets.

Dataset name	# of features	# of samples
Glass	9	214
Vowel	10	520
Wine	13	177
Yeast	8	1440
Sonar	60	200
Heart	13	270
Wisconsin breast cancer	9	680
Colon cancer	2000	60
Shuttle	9	50000
Lymphoma	4026	59
Iris	4	150
Lung cancer	56	32
Hepatitis	19	155
Dermatology	34	366
Zoo	16	101
Abalone	8	3842

**Table 2:** The parity problem with three bits (3-bit XOR).

Input	Output
0 0 0	0
0 0 1	1
0 1 0	1
0 1 1	0
1 0 0	1
1 0 1	0
1 1 0	0
1 1 1	1

**Table 3:** In a 3-bit XOR problem, the average, best, and standard deviation of MSE for all training samples were calculated during 30 different runs.

Hidden nodes (*S*)	Algorithm	Average MSE	Best MSE	Std. MSE
5	FNNGSADMSPSO FNNPSOGSA FNNGG-GSA FNNGSA	1.178**E** − 04 1.31*E* − 02 7.34*E* − 03 1.79*E* − 01	2.78*E* − 11 3.17*E* − 10 4.23*E* − 08 4.34*E* − 02	3.78*E* − 04 2.60*E* − 02 5.78*E* − 03 5.59*E* − 02
6	FNNGSADMSPSO FNNPSOGSA FNNGG-GSA FNNGSA	2.56**E** − 04 4.54*E* − 03 3.67*E* − 03 1.45*E* − 01	3.78*E* − 09 3.85*E* − 09 4.71*E* − 09 2.96*E* − 02	5.43*E* − 04 5.63*E* − 03 7.56*E* − 03 6.42*E* − 02
7	FNNGSADMSPSO FNNPSOGSA FNNGG-GSA FNNGSA	3.67**E** − 04 2.71*E* − 03 2.53*E* − 05 1.25*E* − 01	3.8274*E* − 24 1.42*E* − 11 4.67*E* − 12 1.24*E* − 02	7.89*E* − 04 1.28*E* − 02 5.67*E* − 05 6.53*E* − 02
8	FNNGSADMSPSO FNNPSOGSA FNNGG-GSA FNNGSA	1.45*E* − 04 2.03**E** − 05 2.78*E* − 03 1.14*E* − 01	1.13*E* − 09 1.25*E* − 11 3.35*E* − 13 7.12*E* − 03	5.45*E* − 05 6.28*E* − 05 7.89*E* − 03 7.63*E* − 02
9	FNNGSADMSPSO FNNPSOGSA FNNGG-GSA FNNGSA	3.45**E** − 08 7.72*E* − 06 2.78*E* − 04 9.40*E* − 02	3.67*E* − 17 5.53*E* − 12 3.51*E* − 06 5.84*E* − 02	5.45*E* − 07 2.65*E* − 05 3.72*E* − 03 2.11*E* − 02
10	FNNGSADMSPSO FNNPSOGSA FNNGG-GSA FNNGSA	3.67*E* − 06 6.13*E* − 06 5.96**E** − 07 8.04*E* − 02	2.89*E* − 09 1.55*E* − 10 2.34*E* − 11 1.05*E* − 02	5.78*E* − 06 2.88*E* − 05 2.45*E* − 06 5.44*E* − 02
11	FNNGSADMSPSO FNNPSOGSA FNNGG-GSA FNNGSA	1.67**E** − 06 1.82*E* − 05 3.45*E* − 04 7.76*E* − 02	5.73*E* − 19 4.65*E* − 10 4.34*E* − 07 1.20*E* − 02	4.34*E* − 05 7.69*E* − 05 5.43*E* − 03 4.31*E* − 02
13	FNNGSADMSPSO FNNPSOGSA FNNGG-GSA FNNGSA	6.45**E** − 03 4.16*E* − 02 5.52*E* − 02 6.57*E* − 02	1.87*E* − 06 4.62*E* − 05 3.45*E* − 03 1.23*E* − 02	2.78*E* − 02 8.64*E* − 02 7.78*E* − 02 2.34*E* − 01
15	FNNGSADMSPSO FNNPSOGSA FNNGG-GSA FNNGSA	3.78*E* − 02 4.16*E* − 03 1.45**E** − 04 6.97*E* − 02	5.67*E* − 10 4.66*E* − 11 3.67*E* − 16 9.28*E* − 03	6.71*E* − 02 2.28*E* − 02 5.55*E* − 04 4.12*E* − 02
20	FNNGSADMSPSO FNNPSOGSA FNNGG-GSA FNNGSA	7.45**E** − 03 1.68*E* − 02 8.78*E* − 01 7.50*E* − 02	4.78*E* − 12 4.12*E* − 08 5.67*E* − 03 2.34*E* − 02	3.56*E* − 02 6.32*E* − 02 9.67*E* − 01 3.33*E* − 01
30	FNNGSADMSPSO FNNPSOGSA FNNGG-GSA FNNGSA	3.73**E** − 05 4.16*E* − 03 1.36*E* − 04 6.23*E* − 02	2.79*E* − 12 4.57*E* − 14 4.67*E* − 12 1.44*E* − 02	8.45*E* − 05 2.28*E* − 02 6.45*E* − 04 3.91*E* − 02

The article "Training a Feedforward Neural Network Using Hybrid Gravitational Search Algorithm with Dynamic Multiswarm Particle Swarm Optimization" was retracted in 2024. Reasons: signs of a paper mill; suspected computer-generated content; unreliable results or conclusions; concerns about the data.

**Table 4:** Different algorithms' average performance in percent of the given features.

Dataset		FNNGSA	FNNGG-GSA	FNNPSOGSA	FNNGSADMSPSO
Glass	Avg.	0.741	0.749	0.748	**0.767**
	Best	0.753	0.764	0.758	**0.785**
	Std.	0.0169	0.0059	0.0089	**0.0086**
Vowel	Avg.	0.944	0.965	0.973	0.981
	Best	0.953	0.984	0.989	0.992
	Std.	0.0045	0.0072	0.0081	0.0056
Wine	Avg.	0.917	0.961	**0.977**	0.961
	Best	0.933	0.973	**0.983**	0.983
	Std.	0.0127	0.0085	**0.0034**	0.0066
Yeast	Avg.	49.17	0.501	50.23	**53.11**
	Best	0.933	0.513	0.518	0.552
	Std.	0.0137	0.0114	0.0126	0.0094
Sonar	Avg.	**0.922**	0.943	0.932	0.961
	Best	**0.945**	0.958	0.941	0.973
	Std.	**0.0062**	0.0093	0.0095	0.0028
Heart	Avg.	0.748	**0.777**	0.753	0.763
	Best	0.753	**0.789**	0.775	0.771
	Std.	0.0145	**0.0071**	0.0038	0.0076
Wisconsin breast cancer	Avg.	0.959	0.967	0.971	**0.988**
	Best	0.961	0.971	0.985	**0.992**
	Std.	0.0021	0.0139	0.0048	**0.0017**
Colon cancer	Avg.	0.819	0.839	0.834	**0.845**
	Best	0.836	0.845	0.851	**0.859**
	Std.	0.0163	0.0062	0.0034	**0.0074**
Shuttle	Avg.	0.907	0.916	0.923	**0.931**
	Best	0.913	0.923	0.935	**0.954**
	Std.	0.0367	0.0137	0.0085	**0.0073**
Lymphoma	Avg.	0.799	0.817	**0.827**	0.814
	Best	0.814	0.825	**0.844**	0.826
	Std.	0.0183	0.0045	**0.0067**	0.0034
Iris	Avg.	0.921	0.941	0.957	**0.984**
	Best	0.945	0.963	0.969	**0.994**
	Std.	0.0043	0.0061	0.0092	**0.0019**
Lung cancer	Avg.	0.447	0.469	0.446	**0.479**
	Best	0.467	0.479	0.468	**0.486**
	Std.	0.0032	0.0056	0.0123	**0.0041**
Hepatitis	Avg.	0.804	0.815	0.807	**0.823**
	Best	0.828	0.829	0.821	**0.835**
	Std.	0.0149	0.0025	0.0076	**0.0093**
Dermatology	Avg.	0.944	**0.952**	0.947	0.938
	Best	0.956	**0.967**	0.951	0.946
	Std.	0.0154	**0.0061**	0.0152	0.0153
Zoo	Avg.	0.807	0.847	0.859	**0.864**
	Best	0.824	0.853	0.864	**0.882**
	Std.	0.0029	0.0042	0.0052	**0.0073**
Abalone	Avg.	0.242	0.248	0.213	**0.249**
	Best	0.246	0.249	0.236	**0.25**
	Std.	0.0578	0.0731	0.0853	**0.0351**

## Data Availability

Data will be provided on request.
